# Incidence and Influencing Factors of Chronic Postthoracotomy Pain in Lung Tumor Patients

**DOI:** 10.1155/2022/7584481

**Published:** 2022-02-24

**Authors:** Jing Peng, Zhonghui Wang, Liang Ma, Weihao Ma, Guo Liu, Hui Zhang, Qiongchuan Wang, Bobo Zhu, Li Zhao

**Affiliations:** Department of Anesthesiology, The Third Affiliated Hospital of Kunming Medical University (Yunnan Cancer Hospital), Kinming 650118, Yunnan, China

## Abstract

**Objectives:**

To estimate the incidence of chronic postthoracotomy pain (CPTP) in lung tumor patients and to explore the influencing factors of the intensity of CPTP.

**Methods:**

Lung tumor patients who underwent video-assisted thoracoscopic surgery (VATS) or thoracotomy were consecutively recruited from October 2016 to December 2017 at Yunnan Cancer Hospital. All the eligible patients were interviewed via telephone at the end of the third month after surgeries to identify the presence of CPTP. The potential influencing factors of CPTP, including pre-, intra-, and postoperative variables, were collected from medical records. A cumulative logit regression model was used to identify the independent influencing factors of the intensity of CPTP.

**Results:**

Three hundred and forty-three patients completed a telephone interview. The estimated overall incidence of CPTP was 67.6% (95% of confidence interval, 95% CI: 62.4%, 72.6%) in lung tumor patients; 70.8% (95% CI: 63.8%, 77.1%) in benign patients and 63.5% (95% CI: 55.2%, 71.3%) in malignant patients; and 78.1% (95% CI: 66.0%, 87.5%) in open chest and 65.2% (95% CI: 59.3%, 70.8%) in VATS. Cumulative logit regression models (intensity order, NRS, 0 ⟶ 1–3 ⟶ 4-) revealed independent influencing factors of CPTP to be patients with diabetes (OR = 0.32; 95% CI: 0.14, 0.76), usage of VATS (OR = 0.47; 95% CI: 027, 0.82), and the amount of intraoperative blood loss (OR = 1.09; 95% CI: 1.00, 1.19).

**Conclusions:**

A high incidence of CPTP is detected in lung tumor patients following the thoracic operation. Patients with diabetes and using VATS are the independent protective factors of the intensity of CPTP, and the increasing amount of intraoperative blood loss is an independent risk factor of the intensity of CPTP.

## 1. Background

Lung tumor is one of the common tumors and its incidence increased rapidly in recent years, especially, malignant tumor [1]. At present, thoracic operation that includes thoracotomy and video-assisted thoracoscopic surgery (VATS) is still the main treatment for lung tumors [2, 3]. Despite the effective therapy, chronic postthoracotomy pain (CPTP) which is defined as pain persisting for at least 3 months after thoracic operations is accused of greatly reduced quality of life and increased morbidity [4]. Bayman and Brennan [5] reported that more than half of patients suffered CPTP; thus, it seriously influenced community health. Previous studies [6–10] have found that CPTP was influenced by age, sex, diabetes, properties of tumor, type of surgery, duration of chest tube drainage, and so on; nevertheless, these influencing factors relatively lack repeatability of studies. Although CPTP is one of the great burdens in community health, the mechanism of CPTP is still unknown; hence, the tracing of the predictors or risk factors of CPTP is particularly important for prevention and prediction. Therefore, the aims of this study were to estimate the incidence of CPTP in lung tumor patients and explore the influencing factors of CPTP.

## 2. Methods

### 2.1. Subjects

Lung tumor patients who underwent VATS or thoracotomy were consecutively recruited from October 2016 to December 2017 at Yunnan Cancer Hospital.

Exclusion criteria include the following: (1) age less than 18 years; (2) histories of preoperative chemotherapy, previous thoracic surgery, thoracic trauma, previous chest and back pain, and previous other malignancies; (3) emergent operation; (4) reoperation was performed within 3 months after surgery; (5) postoperative pulmonary infection and surgical site infection; and (6) American Society of Anesthesiologists (ASA) physical status greater than or equal to 3.

All subjects in this study were given verbal informed consent for their participation, and the oral informed consent process was approved by the Research Ethics Committee of the Department of Anesthesiology at Yunnan Cancer Hospital.

### 2.2. Definition

According to the International Association for the Study of Pain (IASP) [11], the CPTP is defined as follows: (1) the pain developed in the operation area or adjacent parts after the operation; (2) the pain lasted for at least three months; (3) the pain which was different from the preoperative pain; and (4) other causes of the pain should be excluded, such as advanced malignant tumor or chronic infection.

### 2.3. Questionnaire Design and Telephone Interview

All the eligible patients were interviewed via telephone at the end of the third month after surgeries; therefore, this study was conducted from January 2017 to April 2018. The telephone interviews were conducted by well-trained research team members to collect information of CPTP following appointments.

According to the literature review and expert consultation, the data of demographic, pre-, intra-, and postoperative variables were designed into a questionnaire and then collected from the medical record after the consent of the patient.

The most critical aspect of this questionnaire is to identify patients who had really experienced CPTP based on their responses to questions as follows:

1. ‘‘Have you experienced any pain along the scar after surgery, different from what you had before the surgery?”
2. ‘‘Has the pain persisted for at least 3 months?”

If a participant answered “yes” for the presence of pain, patients were then further asked to report the severity of their CPTP by the numerical rating scale (NRS) method as well as the ID pain questionnaire [12], which is used to identify neuropathic pain in CPTP patients.

### 2.4. Surgery, Anesthesia, and Postoperative Pain Management

Two different surgical teams were involved in this study, with both thoracotomy and VATS. The thoracotomy approach used a conventionally lateral or posterior-lateral incision without rib resection during the operation. The skin incision was parallel to the ribs at the intercostal space. Chest tubes (JINGLE®, China, 26-Fr, Disposable Drainage Tube, and DIALL®) were placed before closing the chest, and extreme precautions were used to avoid the injury of intercostal nerves. The VATS approach used a uniform anterior single- or three-port technique with standardized port placements regardless of the lobe to be resected or not. For the single-hole operation, the hole was made in the 5th or 4th intercostal space at the anterior axillary line, while the three holes were located at the 3rd , 7th, and 9th intercostal space at the anterior, middle, and posterior axillary lines, respectively. At the end of the surgery, two chest tubes were inserted just similar to thoracotomy. The draining chest tube was removed as soon as no air leakage was detected for more than 24 hours, the total amount of pleural effusion was less than 200 ml per day, and no chylothorax or bleeding was present.

A total intravenous anesthesia (TIVA) technique composed of midazolam, propofol, sufentanil, and remifentanil, and intermittent rocuronium was used to maintain adequate anesthesia after induction. No paravertebral or epidural block was administered pre- or postoperatively. The postoperative pain management of all patients was patient-controlled infusion pump (PCIA), involving a programme to deliver a total of 100 ml of the mixture of sufentanil, dextrozine, ondansetron, and saline within 48 hours with a continuous dose of 1-2 micrograms per hour, along with patient-controlled bolus of 2-3 micrograms at a lockout interval of 10 minutes. The bolus dosage was subsequently adjusted and titrated for optimal analgesia (visual analogue scale (VAS) score less than 3). The patients' pain status was managed by a dedicated Acute Pain Service (APS) team from the Department of Anesthesiology and assessed on the third day after surgery.

### 2.5. Analysis

Demographic, pre-, intra-, and postoperative variables were compared across the 3 levels of intensity of CPTP using the Kruskal–Wallis test. Based on the results of univariate analyses, variables were selected for inclusion in initial cumulative logit regression models to identify the independent influencing factors of CPTP intensity. Model refinement was conducted using manual backward exclusion, sequentially removing variables not contributing significantly to the fit of the model based on the change in log-likelihood of successive models. All the significance tests were two-sided, and *P* values less than 0.05 were considered statistical significance.

## 3. Results

Three hundred and seventy-nine lung tumor patients who underwent thoracic surgery were recruited in this study; thirty-five patients were lost to follow-up and one patient died. The remaining 343 patients finished the telephone interview, giving a completion rate of 90%. Among these 343 patients, 232 were diagnosed as CPTP, and thus, the estimated overall incidence of CPTP was 67.6% (95% of confidence interval, 95% CI: 62.4%, 72.6%) in the whole study sample; 78.1% (95% CI: 66.0%, 87.5%) in open chest and 65.2% (95% CI: 59.3%, 70.8%) in VATS; and 70.8% (95% CI: 63.8%, 77.1%) in benign patients and 63.5% (95% CI: 55.2%, 71.3%) in malignant patients; however, neither types of surgery (*P* = 0.393) nor the properties of tumor (*P* = 0.155) differed significantly. Furthermore, among 232 CPTP patients, 148 patients (63.8% (95% CI: 57.2%, 70.0%)) were identified as neuropathic pain in the current study.

Figure 1 shows the distribution of NRS among CPTP patients, and most of them were less than 5. On the basis of the NRS distribution, the intensity of CPTP was defined as mild (NRS = 1–3) and moderate or severe (NRS = 4 and above, 4-), as well as non-CPTP (NRS = 0) in this study.

Table 1 shows the general characteristics of patients according to the 3 levels of NRS. Sex, age, height, weight, smoking, and drinking showed no significant difference across the levels.  Figure 2 compares the distribution of the properties of tumor across the 3 levels; similar to general characteristics, the difference was without significance.

Pre-, intra-, and postoperative variables are shown in Table 2. In this study, the percentages of non-CPTP patients suffering from diabetes and hypertension were relatively higher than those of CPTP patients. Moreover, the usage of VATS significantly differed across the 3 levels of NRS. In Figure 3, the CPTP groups relatively had higher proportions of using spreader than non-CPTP group; however, the using time of spreader among the 3 groups did not show significant difference.

Table 2 also shows the patients' ASA physical status ranged from I to II, and no significant difference was found among the 3 groups. Similarly, type of procedure, intraoperative intercostal nerve block, postoperative hospital stays, postoperative morphine use, duration of drainage, and postoperative antibiotic use also showed nonsignificant difference across the 3 groups. The values of preoperative albumin, duration of surgery, dosage of sufentanil, and intraoperative blood loss relatively differed (0.05 < *P* < 0.10) among the 3 groups.

On the basis of the results of the univariate analyses, sex, age, height, weight, preoperative albumin, history of diabetes and hypertension, usage of VATS, duration of surgery, usage of spreader, duration of using spreader, dosage of sufentanil, and intraoperative blood loss were included in an initial cumulative logit model to identify the independent influencing factors of the intensity of CPTP (intensity order, NRS, 0 ⟶ 1–3 ⟶ 4-). After model refinement, the history of diabetes, usage of VATS, and intraoperative blood loss remained.  Table 3 shows the patients with diabetes (OR = 0.32, 95% CI: 0.14, 0.76) and usage of VATS (OR = 0.47, 95% CI: 027, 0.82) favored a lower intensity of CPTP, whereas more intraoperative blood loss (OR = 1.09, 95% CI: 1.00, 1.19) favored a higher intensity of CPTP.

## 4. Discussion

In this study, the incidence of CPTP was estimated to be 67.6% in Chinese lung tumor patients after thoracic surgery, 70.8% in benign patients, and 63.5% in malignant patients. Patients with diabetes and the use of VATS could reduce the intensity of CPTP; by contrast, the increasing amount of intraoperative blood loss could increase it.

CPTP is a highly prevalent complication following thoracic surgery. The incidence of CPTP has been investigated for decades and has been estimated between 8% and over 80% [8, 9, 13–17]. One difficulty arises in comparing the incidence of CPTP among related studies because of different definitions used. Two previous studies were conducted in the United States [18] and China [8]. The United States study estimated the incidence of CPTP at 3 months to be 34.3% which is noticeably lower than the current study result; however, the Chinese study reported the incidence of 64.5% which is similar to this study. This might be due to the different definitions of pain between the two previous studies. In the Chinese study, patients reported persistent and intense discomfort after surgery, such as acid distension and anesthesia, which was judged as pain, which was analogue to our study and might differ from the study in the United States.

An additional lack of comparability arises from the types of patients and surgeries employed. A study conducted in Korea [15] reported an incidence of CPTP in patients with traumatic multiple rib fractures of 52.3%. Moreover, a previous study [19] found that of 27% in patients after VATS. Regardless of the different definitions and types of patients, Bayman and Brennan [5] conducted a systematic review and demonstrated that the incidence of CPTP just following thoracotomy was 58% (ranged from 31% to 96%) at 3 months, which is slightly lower than current study result. However, Kinney et al. [10] estimated a rate of CPTP of 68% in patients who underwent thoracotomy, which was similar to our result although VATS and thoracotomy were both employed in the current study. This phenomenon indicates the complexity of the incidence of CPTP, which may be influenced by not only types of patients and surgeries but also some potential factors such as cultures [20] or pain management [21].

An interesting finding of the current study is that patients with diabetes were identified as an independent protective factor of CPTP by multivariate model. According to our literature review, numerous researches have studied on CPTP or diabetes; however, only few studies [6, 8, 17] reported the association between CPTP and diabetes. Wang et al. [8] and Kar et al. [6] found that patients with diabetes was an independent risk factor of CPTP which was contrary to the finding of this study. This dilemma might be explained by the aspects of diabetic patients. As known that diabetic peripheral neuropathy (DPN) is one of the complications of diabetes as well as painful diabetic peripheral neuropathy (PDPN) and non-PDPN, the mechanisms of DPN and PDPNs are still unknown [22–25]. Nevertheless, the pain sensory of patients with neuropathy may be classified into 3 patterns, namely, positive pattern, negative pattern, and no symptoms at all. [23]. The positive pattern indicates increased sensory perception, which could explain the reason diabetes is the risk factor of CPTP. Thus, the protective effect on CPTP of diabetes could be due to the negative pattern which means numbness or sensory loss. Another point worth noting is that, in our univariate analysis, the patient with hypertension was also a significant protective factor of CPTP, which is similar to a previous study [17], although it was removed from the final cumulative logit model because of nonsignificance. Furthermore, Sacco et al. [26] reported that, with the progress of hypertension, the pain sensory would increase first and then decrease in patients suffering from chronic pain. This phenomenon might suggest another potential explanation of the effect of diabetes on CPTP.

VATS is an alternative approach for lung surgery which is considered to be less tissue trauma and shorter recovery [27–31]. VATS as a minimally invasive approach is expected to reduce postoperative pain; however, the relationship between VATS and CPTP is still ambiguous. Some of the relative studies reported that the rates of CPTP in VATS and thoracotomy showed no difference [32–35], and meanwhile, others [16, 30, 31, 36] found that VATS was a protective factor of CPTP, which is consistent with our result. One of the reasons for the different conclusions might be due to the time of interview at different postoperative days. A nonsignificant result study interviewed patients at an average of 22 months after surgeries [32], compared with others ranging from 3 [31] to 12 [30] months. This phenomenon might suggest that, with the recovery process, the differences in the rate of CPTP at VATS and thoracotomy are elapsing. Other reasons might be the different types of patients and sample size of the study.

Under the control of 12 pre-, intra-, and postoperative variables, the increasing amount of intraoperative blood loss is identified as an independent risk factor of the intensity of CPTP, which indicates that no matter VATS or thoracotomy, decreasing the amount of intraoperative blood loss would relief the chronic postoperative pain. Similarly with this study, Homma et al. [7] detected intraoperative blood loss was a risk factor of neuropathic pain via univariate analysis, but it was subsequently removed because of nonsignificance in the final logistic regression model. In Homma's study, patients were classified based on neuropathic pain and nonneuropathic pain which differed from ours which allocated patients into pain and nonpain without the discrimination of the type of pain. Thus, the nonneuropathic pain group might include the patients who were suffering from chronic pain but not neuropathic pain, which would reduce the statistical efficiency of identifying differences between two groups, especially, when intraoperative blood loss is a nonspecified influencing factor of neuropathic pain. This phenomenon hints that the CPTP including both neuropathic pain and nonneuropathic pain may be related to oxidative stress response through ischemia-reperfusion which is caused by intraoperative blood loss of thoracic operation. Unfortunately, we are not able to test the related inflammatory factors to explore the changes between CPTP and non-CPTP because of the study design; thus, further study is suggested.

This study has several limitations. Firstly, because of the study design, we are not able to further explain the mechanisms of the relationships between CPTP and diabetes and intraoperative blood loss. Secondly, the postoperative acute pain is absent in this study because all patients were evaluated on the third day after surgery, and this may not necessarily represent the actual pain level of patients. Thirdly, this is a single-center study, and additional data from multicenter studies will be needed to verify our findings. Additionally, the employment of the surgical approach, VATS or thoracotomy, is based on the therapy guidelines; therefore, the selection bias may occur in this study.

In conclusion, this study demonstrated the incidence of CPTP was 67.6% in lung tumor patients, 70.8% in benign patients, and 63.5% in malignant patients. Under the control of pre-, intra- and postoperative variables, patients with diabetes (OR = 0.32; 95% CI: 0.14, 0.76) and using VATS (OR = 0.47; 95% CI: 027, 0.82) are independent protective factors of the intensity of CPTP, and the increasing amount of intraoperative blood loss (OR = 1.09; 95% CI: 1.00, 1.19) is an independent risk factor of the intensity of CPTP. Considering the high incidence of CPTP in the community, the related departments need to increase policy support in both physical and physiological aspects, especially for patients with risk factors.

## Figures and Tables

**Figure 1:** Distribution of NRS among CPTP patients. CPTP, chronic postthoracotomy pain; NRS, numerical rating scale.

**Figure 2:** Distribution of the properties of tumor across the 3 levels of NRS among lung tumor patients. Notes: *P* = 0.147, the result of Kruskal–Wallis test. NRS, numerical rating scale.

**Figure 3:** Distribution of the using time of spreader across 3 levels of NRS among lung tumor patients (*n* = 66). Notes: *P* = 0.106, the result of Kruskal–Wallis test. Abbreviations: NRS, numerical rating scale.

**Table 1:** The general characteristics of lung tumor patients with thoracic surgery according to the three levels of NRS scores.

Items	0, *n* = 111	1–3, *n* = 169	4–, *n* = 63	*P*
Sex				0.904
Male	63 (56.8)	99 (58.6)	35 (55.6)	
Female	48 (43.2)	70 (41.4)	28 (44.4)	
Age (years)	53.59 ± 9.76	51.65 ± 10.62	53.79 ± 11.91	0.149
Height (cm)	163.56 ± 6.91	164.06 ± 7.96	162.05 ± 6.04	0.130
Weight (kg)	61.85 ± 9.94	62.01 ± 10.56	60.59 ± 11.23	0.445
BMI	23.22 ± 3.73	23.02 ± 3.21	23.09 ± 3.69	
Educated				0.121
No	50 (45.0)	96 (56.8)	36 (57.1)	
Yes	61 (55.0)	73 (43.2)	27 (42.9)	
Smoking				0.636
No	69 (62.2)	112 (66.3)	38 (60.3)	
Yes	42 (37.8)	57 (33.7)	25 (39.7)	
Drinking				0.705
No	90 (81.1)	134 (79.3)	53 (84.1)	
Yes	21 (18.9)	35 (20.7)	10 (15.9)	
Surgical history				0.722
No	83 (74.8)	120 (71.0)	44 (69.8)	
Yes	28 (25.2)	49 (29.0)	19 (30.2)	

Notes: continuous variables are presented as the mean and the standard deviation, mean ± sd. Categorical variables are presented as the number, with the percentage in parentheses, frequency (%). NRS, numerical rating scale.

**Table 2:** The perioperative information of lung tumor patients with thoracic surgery according to the three levels of NRS scores.

Items	0, *n* = 111	1–3, *n* = 169	4–, *n* = 63	*P*
ASA physical status				0.212
I	60 (54.1)	109 (64.5)	37 (58.7)	
II	51 (45.9)	60 (35.5)	26 (41.3)	
Preoperative albumin (g)	46.55 ± 3.53	46.08 ± 4.17	45.03 ± 4.26	0.075
History of diabetes				0.007
No	96 (86.5)	163 (96.4)	59(93.7)	
Yes	15 (13.5)	6 (3.6)	4 (6.3)	
History of hypertension				0.028
No	90 (81.1)	155 (91.7)	53 (84.1)	
Yes	21 (18.9)	14 (8.3)	10 (15.9)	
Type of surgery				0.419
Wedge excision	30 (27.0)	60 (35.5)	17 (27.0)	
Lobectomy	74 (66.7)	93 (55.0)	39 (61.9)	
Others	7 (6.3)	16 (9.5)	7 (11.1)	
VATS				0.003
No	14 (12.6)	29 (17.2)	21 (33.3)	
Yes	97 (87.4)	140 (82.8)	42 (66.7)	
Duration of surgery (≥4 hrs)				0.096
No	95 (85.6)	130 (76.9)	46 (73.0)	
Yes	16 (14.4)	39 (23.1)	17 (27.0)	
Use of spreader				0.013
No	96 (86.5)	138 (81.7)	43 (68.3)	
Yes	15 (13.5)	31 (18.3)	20 (31.7)	
Intraoperative blood loss (100 ml)^*∗*^	1.00 (1.00)	1.00 (1.00)	1.00 (1.50)	0.073
Sufentanil (mg)^*∗*^	0.04 (0.02)	0.04 (0.02)	0.03 (0.02)	0.068
Remifentanil (mg)^*∗*^	1.50 (0.75)	1.50 (1.00)	1.50 (0.85)	0.308
Intercostal nerve block				0.929
No	99 (89.2)	150(88.8)	55 (87.3)	
Yes	12 (10.8)	19 (11.2)	8 (12.7)	
Postoperative hospital stay (days)	8.56 ± 3.67	8.08 ± 2.57	8.43 ± 3.34	0.657
Postoperative morphine use (times)^*∗*^	0 (1.00)	0 (1.00)	0 (1.00)	0.115
Duration of drainage (≥4 days)				0.428
No	72 (64.9)	112 (66.3)	36 (51.7)	
Yes	39 (35.1)	57 (33.7)	27 (42.9)	
Postoperative antibiotic use (days)	6.37 ± 2.48	6.08 ± 2.26	6.62 ± 3.18	0.499

Notes: continuous variables are presented as the mean and the standard deviation, mean ± sd. Categorical variables are presented as the number, with the percentage in parentheses, frequency (%). ^*∗*^median (interquartile range, IQR). NRS, numerical rating scale; ASA, American Society of Anesthesiologists; VATS, video-assisted thoracoscopic surgery.

**Table 3:** Cumulative logit regression results of intensity of CPTP influencing factors in lung tumor patients following thoracic surgery.

Items	Coefficient	Ordinal OR (95% CI)	*P*
History of diabetes	−1.138	0.32(0.14, 0.76)	0.009
VATS	−0.755	0.47(0.27, 0.82)	0.008
Intraoperative blood loss (100 ml)	0.089	1.09(1.00, 1.19)	0.044

Notes: intensity CPTP order: NRS 0 < 1–3 < 4. Independent variables of baseline initially were included in the model but subsequently removed because of nonsignificance: sex, age, height, weight, preoperative albumin, history of hypertension, duration of surgery, usage of spreader, duration of using spreader and dosage of sufentanil. CPTP, chronic postthoracotomy pain; VATS, video-assisted thoracoscopic surgery; OR, odds ratio; 95% CI, 95% of confidence interval.

## Data Availability

The datasets used and analyzed during the current study are available from the corresponding author upon reasonable request.
